# The Effect of Azithromycin Combined with Palm Massage on Pulmonary Function of Children with Mycoplasma Pneumonia

**DOI:** 10.1155/2022/1857055

**Published:** 2022-07-04

**Authors:** Haiyan Li, Dandan Xu

**Affiliations:** Department of Respiratory, Maternal and Child Health Hospital of Jiujiang City, Jiujiang, Jiangxi, China

## Abstract

**Objective:**

The study aimed to determine the effect of azithromycin combined with palm massage on the pulmonary function of children suffering from mycoplasma pneumonia, as well as associated complications.

**Methods:**

A total of 60 cases of children suffering from mycoplasma pneumonia admitted to our hospital from May 2018 to May 2020 were selected as study subjects and assigned to either the observation group or the control group. Lung function indices and changes in the levels of inflammatory markers were measured before and after treatment in both groups, and the results were compared to assess treatment efficacy.

**Results:**

There was no statistically significant difference in lung function indices between the two groups before treatment (*P* > 0.05), while there was a statistically significant difference between the two groups after treatment (*P* < 0.05), with the observation group outperforming the control group. Similarly, there was no statistically significant difference in the levels of such inflammatory markers as IL-6 and TNF-*α* between the two groups before treatment (*P* > 0.05). After treatment, there was a decrease in the levels of inflammatory markers in both groups, but a much larger decrease was seen in the observation group (*P* < 0.05) than in the control group. The total treatment efficacy in the observation group was 93.3%, which was significantly higher than that of 70.0% in the control group (*P* < 0.05).

**Conclusion:**

The application of palm massage combined with azithromycin in the treatment of children suffering from mycoplasma pneumonia produces outstanding results in terms of relieving symptoms and improving pulmonary function.

## 1. Introduction

Mycoplasma pneumonia is a common respiratory infection among children and young adults that is caused by *Mycoplasma pneumoniae*, a strict human pathogen that adheres to the respiratory epithelium by means of a specialized attachment structure. It accounts for 10% to 20% of all cases of pneumonia. Clinical manifestations include fever of varying degrees, dyspnea, and cough. It has an obvious seasonal variation, being proportionately more common during the winter and spring and follows a long disease course that may progress rapidly. Disease progression usually takes the form of involvement of multiple extrapulmonary sites, with the CNS involvement being particularly serious, or may take the form of development into bronchial asthma [1], which further complicates clinical management. Children are especially susceptible to mycoplasma pneumonia due to underdeveloped organs and a relatively weak immune system in this group of patients. Current treatment of mycoplasma pneumonia mainly relies on the use of azithromycin. Azithromycin is a semisynthetic derivative of erythromycin, a drug that belongs to a class of antibiotics known as macrolides that mainly work by inhibiting the formation of the bacterial 50 S ribosomal subunit and are active against susceptible Gram-positive, atypical, and a few Gram-negative organisms. The drug is highly active against *M. pneumoniae*, the causative agent of mycoplasma pneumonia. However, the widespread use of azithromycin has been accompanied by the emergence of certain strains of *M. pneumoniae* that are resistant to the drug, and there are cases where monotherapy fails to produce the desired effect. Also, azithromycin is not exempt from the toxic side effects of western drugs, which are associated with an increased incidence of complications such as discomfort to the gastrointestinal tract in children, and it is prone to drug resistance. Thus, coupled with the young age of most of the patients suffering from mycoplasma pneumonia, as well as their poor adherence to treatment, usually results in reduced efficacy of the drug [2]. Traditional Chinese medicine (TCM) has accumulated a very rich experience in the treatment of mycoplasma pneumonia. In TCM, the disease is believed to be secondary to the impact of external factors such as wind, cold, and heat, and the treatment focuses on the regulation of qi and blood, relaxation of tendons and collaterals, and maintenance of the balance of yin and yang. In view of this, this study adopted the TCM method of treating mycoplasma pneumonia by palm massage and combined it with usage of azithromycin to determine the treatment efficacy of this approach. A total of 60 cases of mycoplasma pneumonia in our hospital were included in the study from May 2018 to May 2020.

## 2. Materials and Methods

### 2.1. General Information

Sixty cases of children suffering from mycoplasma pneumonia admitted to our hospital from May 2018 to May 2020 were selected as study subjects and were assigned to either the observation group or the control group, according to odd and even numbers placed randomly in an envelope. Each group comprised 30 cases. There were 16 males and 14 females in the observation group, with a mean age of (4.59 ± 1.32) years (9 months to 8 years) and a mean duration of disease of (6.35 ± 1.16) days (2 to 10 days). There were 17 males and 13 females in the control group, with a mean age of (4.51 ± 1.27) years (7 months to 8 years) and a mean duration of illness of (6.32 ± 1.13) days (1 to 11 days). The two groups were comparable in terms of general information (*P* > 0.05). The guardians of the children involved in this study were fully informed of the purpose and method of this study, and all of them signed the informed consent form. This study was also reviewed and approved by the medical ethics committee of our hospital.

### 2.2. Inclusion and Exclusion Criteria

Children that met the following criteria were included in the study:

1. Children who were diagnosed with mycoplasma pneumonia by chest X-ray and CT [3]
2. Children with symptoms such as cough and fever
3. Children who tested for a positive antibody against *Mycoplasma pneumonia*
4. Children with complete clinical data

Children that met the following criteria were excluded from the study:

1. Children with vital organ damage
2. Children with mental abnormalities, or those who were unconscious
3. Children with cancer
4. Children with other respiratory diseases
5. Children who could not cooperate with or voluntarily withdrew from the study
6. Children with a history of allergy or intolerance to the drugs used in this study
7. Children with a weak immune system or coagulation disorders
8. Children with combined systemic infections
9. Children who could not tolerate palm massage therapy

### 2.3. Methods

After admission, the children underwent routine examination and a diagnosis was performed. This was followed by symptomatic treatment, which included cough suppression, control of infection, nutritional support, maintenance of airway patency, and oxygenation if necessary. Patients in the control group were treated with azithromycin alone. Azithromycin (10 mg/kg) was diluted in 5% dextrose solution and given intravenously at a dosage of ≤500 mg. The drug was given one time per day, for a total of 5 days. Subsequently, the route of administration was switched to the oral route. The patients were treated for a total of 2 weeks. Patients in the observation group were treated with a combination of azithromycin and palm massage. The palm massage procedures are as follows:

1. Clearing the lung meridian: the massage therapist holds the child's hand in the left hand, keeping the child's fingers upward and outward and uses the right thumb and the palm to massage the child's ring finger from bottom to top, repeating the procedure about 100∼300 times.
2. Shunyun Bagua (clockwise palm massage): with the child in the guardian's arms, the therapist holds the child's left hand, keeping the palm facing upward and uses the thumb to massage the child's palm in a clockwise direction, starting from the Qian Diagram to the Kan Diagram and through to the Dui Diagram in the Bagua Diagrams of the palm, repeating the procedure about 100∼200 times.
3. Feijing Zouqi method: the therapist holds the child's hand in the left hand, presses the Quchi acupoint, and then presses the Yin chi and Yang chi acupoints with the thumb and the middle finger while keeping the fingers pointing upward and outward, repeating the procedure about 50∼100 times.
4. Thenar eminence and hypothenar eminence massage: the therapist uses the left thumb to gently push the thenar eminence of the thumb, from the proximal to the distal end about 20 times and then reverses the direction of motion. The same method is used to massage the hypothenar eminence.

### 2.4. Observational Indicators

The treatment was evaluated by recording the time taken for symptoms to disappear, duration of hospitalization, lung function indices, levels of inflammatory markers, and presence or absence of complications:

1. 5 ml of peripheral venous blood was collected and centrifuged at 3000 r/min for 10 min to isolate the serum. Serum TNF-*α* and IL-6 levels were then determined using the ELISA, with the kits being provided by Chengdu Super Nine Eight Biotechnology Co. Ltd.
2. Lung function indices were determined using the FGC-A + Anke spirometer, which was provided by Jinan Hao Lai Bao Medical Equipment Co. Ltd.
3. Evaluation criteria: treatment was considered to be markedly effective if all related clinical indices returned to normal and symptoms disappeared after treatment. It was considered to be effective if symptoms were relieved, and the level of inflammatory markers decreased to a certain extent. If there was no significant improvement in symptoms or if symptoms deteriorated, then the treatment was considered to be ineffective. The total treatment efficacy is the sum of the number of cases in which treatment was markedly effective and cases in which treatment was effective, which was expressed as a percentage of the total number of cases that were treated [4].

### 2.5. Statistical Methods

Statistical analysis of the data was performed using the SPSS22.0 software. The count data were expressed as (%) using the chi-square test, and the measurement data were expressed as ($\bar{x}\pm s$) using the *t*-test. *P* < 0.05 was considered statistically significant.

## 3. Results

### 3.1. Time Taken for Symptoms to Disappear

The time taken for symptoms such as fever, cough, and rales to disappear, as well as the duration of hospital stay was recorded and compared. It was found that these times were significantly shorter in the observation group than in the control group (*P* < 0.05) ( see Table 1 for illustration).

### 3.2. Lung Function Indices

There was no statistically significant difference in lung function indices between the two groups before treatment (*P* > 0.05). After treatment, lung function indices were significantly better in the observation group than in the control group (*P* < 0.05) (see Table 2 for illustration).

### 3.3. Inflammatory Markers

There was no statistically significant difference in the levels of IL-6 and TNF-*α* between the two groups before treatment (*P* > 0.05). After treatment, the levels of both inflammatory markers decreased in both groups. However, a much larger decrease was seen in the observation group than in the control group (*P* < 0.05) (see Table 3 for illustration).

### 3.4. Treatment Efficacy

Treatment was considered to be markedly effective in 21 cases and was considered to be effective in 7 cases in the observation group. This translates to a total treatment efficacy of 93.3%. In the control group, treatment was considered to be markedly effective in 15 cases and was considered to be effective in 6 cases, translating to a total treatment efficacy of 70.0%. This shows that the total treatment efficacy in the observation group was significantly higher than that in the control group (*P* < 0.05) (see Table 4 for illustration).

### 3.5. Incidence of Complications

The observation group had 1 case of nausea and vomiting and 1 case of dizziness, translating to an incidence of complications of 6.7%. The control group had 2 cases of nausea and vomiting, 1 case of diarrhea, 3 cases of dizziness, and 2 cases of pruritus, translating to an incidence of complications of 26.7%. The incidence of complications in the observation group was significantly lower than that in the control group (*P* < 0.05) (see Table 5 for illustration).

## 4. Discussion

The study found that the time taken for symptoms to disappear was significantly shorter in the observation group than in the control group, indicating that palm massage was able to accelerate the recovery process.

Palm massage relies heavily on the principles of meridians, internal organs, and the five elements. It follows the circulation of qi and blood, which facilitates the flow of qi and blood while unblocking the meridians and maintaining the balance of internal organs [5]. Palm massage regulates the functions of the internal organs of the whole body, and light pushing on the palm of the child at the appropriate location promotes the flow of qi and blood and harmonizes the balance of yin and yang [6]. Clearing the lung meridian improves pulmonary circulation and ventilation, significantly improving symptoms [7]. Shunyun Bagua was conventionally used in the treatment of diarrhea, and its application in mycoplasma pneumonia is effective in relieving cough and regulating qi. Feijing Zouqi massage relieves cough and chest tightness. Thenar eminence and hypothenar eminence massage improves blood circulation, pulmonary function, and enhances immunity [8, 9].

The patients in the observation group showed significant improvement in all lung function indices after treatment, and the improvement outstripped that was seen in the control group. The previous research study suggests that the inflammatory markers IL-6 and TNF-*α* may play a role in the pathogenesis of pediatric mycoplasma pneumonia. Moreover, microbial invasion of the body results in tissue damage, which then leads to secretion and overexpression of inflammatory markers [5]. In this study, the levels of inflammatory markers reduced in both groups following treatment, but a more pronounced reduction was seen in the observation group. The possible mechanism is that Th1 and Th2 cells can produce inflammatory cytokines such as IFN-*γ*, TNF-*α,* and IL-4 and mediate cellular and humoral immune responses, and mycoplasma pneumonia can cause abnormal differentiation of T lymphocyte subsets in children with elevated levels of IFN-*γ*, TNF-*α*, IL-4, and Th1/Th2 as the main manifestations. And macrolide antibiotics can block transpeptidase and exert an antibacterial effect by inhibiting protein synthesis in Mycoplasma *pneumoniae*. The total treatment efficacy in the observational group was 93.3%, compared to 70.0% in the control group. This suggests that the combination of azithromycin and palm massage is more effective than monotherapy using azithromycin alone. The follow-up results showed that there was a lower incidence of complications in the observation group than in the control group, suggesting that the combination of azithromycin and palm massage minimizes the side effects of azithromycin and improves the overall prognosis.

### 4.1. Limitations

The limitations of this study include the short duration of the study, the small sample size, and the relatively narrow observation parameters. Further studies with longer durations, larger sample sizes, and longer follow-up periods may need to be conducted to arrive at a more definite conclusion.

## 5. Conclusion

In conclusion, the combination of azithromycin and palm massage in the treatment of children with mycoplasma pneumonia is more effective than monotherapy with azithromycin alone. It accelerates symptom relief and profoundly reduces the levels of inflammatory markers and is associated with a lower incidence of complications. It is an approach that must be used whenever possible and that deserves more widespread application.

## Figures and Tables

**Table 1:** Comparison of the time taken for symptoms to disappear and hospitalization time (*d*, $\bar{x}\pm s$).

Group	*n*	Fever	Cough	Rales	Hospitalization time
Observation group	30	2.12 ± 0.32	5.48 ± 1.21	5.82 ± 1.21	9.34 ± 1.24
Control group	30	3.39 ± 0.14	7.23 ± 1.83	7.28 ± 1.24	12.38 ± 2.16
*T*	*—*	19.915	4.369	4.616	6.685
*P*	*—*	≤0.001	≤0.001	≤0.001	≤0.001

**Table 2:** Comparison of lung function indices ($\bar{x}\pm s$).

Group		FVC (L)	FEV1 (L)	FEV1/FVC (%)
Observation group (*n* = 30)	Before treatment	1.85 ± 0.23	1.38 ± 0.42	52.32 ± 4.22
	After treatment	3.04 ± 0.52^*∗*^	1.97 ± 0.34^*∗*^	75.59 ± 4.14^*∗*^
	*t*	11.463	5.980	21.560
	*P*	≤0.001	≤0.001	≤0.001

Control group (*n* = 30)	Before treatment	1.83 ± 0.18	1.38 ± 0.49	52.31 ± 4.24
	After treatment	2.35 ± 0.52	1.66 ± 0.36	63.94 ± 4.22
	*T*	5.176	2.522	10.648
	*P*	≤0.001	≤0.001	≤0.001

**Table 3:** Comparison of inflammatory marker levels ($\bar{x}\pm s$).

Groups	*n*	IL-6 (ng/L)		TNF-*α* (ng/L)	
		Before treatment	After treatment	Before treatment	After treatment
Observation group	30	46.14 ± 6.73	18.42 ± 2.04^*∗*^	43.26 ± 4.04	21.05 ± 2.15^*∗*^
Control group	30	46.24 ± 6.59	29.16 ± 3.46^*∗*^	43.37 ± 4.18	30.54 ± 3.36^*∗*^
*T*	—	0.058	14.646	0.104	13.031
*P*	—	0.954	≤0.001	0.918	≤0.001

Note: compared to the control group after treatment, *∗P* < 0.05.

**Table 4:** Comparison of the total treatment efficacy (%).

Groups	*n*	Markedly effective	Effective	Ineffective	Total efficacy (%)
Observation group	30	21 (70.0)	7 (23.3)	2 (6.7)	28 (93.3)
Control group	30	15 (50.0)	6 (20.0)	9 (30.0)	21 (70.0)
*X* ^2^	—	—	—	—	5.455
*P*	—	—	—	—	0.020

**Table 5:** Comparison of the incidence of complications (%).

Groups	*n*	Nausea and vomiting	Diarrhea	Dizziness	Pruritus	Incidence of complications (%)
Observation group	30	1 (3.3)	0 (0.0)	1 (3.3)	0 (0.0)	2 (6.7)
Control group	30	2 (6.7)	1 (3.3)	3 (10.0)	2 (6.7)	8 (26.7)
*X* ^2^	—	—	—	—	—	4.320
*P*	—	—	—	—	—	0.038

## Data Availability

The datasets used and analysed during the current study are available from the corresponding author on reasonable request.
